This article has been retracted.

# An Intervention Study on Children's Healthy Joint Attention Skills Based on a Mixed Instructional Approach of DTT and PRT

**DOI:** 10.1155/2022/5987582

**Published:** 2022-03-18

**Authors:** Shengmin Liu, Shufang Mao

**Affiliations:** ^1^Department of Psychology, School of Teacher Education, Huzhou University, Huzhou, Zhejiang 313000, China; ^2^Mental Health Education and Guidance Center, Zhejiang Financial College, Hangzhou, Zhejiang 310018, China

## Abstract

Joint attention is an important element that influences children's early development of communication and sociality, and joint attention is more often than not the earliest incipient of their prosocial behavior. Joint attention skills are one of the core deficits of children with autism, and identifying and remediating the core problems of autism is a popular area of interest, with joint attention being the focus of attention. The aim of this study was to investigate whether the combined orientation model of Discrete Trial Teaching (DTT) and Pivotal Response Training (PRT) could improve the joint attention skills of children with autism. This study used a cross-behavioral multitest design in a single-subject study with two preschool children with autism as subjects, with the independent variable being joint attention teaching and the dependent variable being the three joint attention skills (eye gaze, following directions, and active display). After the instructional intervention, children with autism showed a significant increase in the correctness of “eye alternation,” “following directions,” and “moving displays.”

## 1. Introduction

Joint attention is considered to be the basis for higher level cognitive and social skills such as theory of mind. When children are able to use outward behavior or verbal expressions to get the attention of others and share their interests and experience of things (people, events, and objects), this means that the child is developing joint attention well [1]. In developing a theory of mind and language, joint attention becomes one of the core skills necessary for children with autism [2].

The lack of joint attention seriously affects the acquisition of language expression and social skills in children with autism [3]. The deficits in language expression and social skills can place children with autism in a closed environment, and this situation can have a negative impact on their personality development and psychophysical health development and predispose them to behavioural problems [4]. Delayed joint attention development is evident and widespread in children with autism at an early age. Joint attention is a foundation for the development of language and interpersonal interactions and is therefore there is an urgent need for effective follow-up treatment of children with autism.

As joint attention is a foundation for the development of language and interpersonal interaction, it has important links with communication skills, social skills, emotional regulation, and play [5]. Therefore, improving the joint attention of children with autism can help improve the development of nonverbal and verbal expression, as well as social initiative and emotional control in children with autism. In recent years, many studies have shown that coattentive teaching can improve the coattentive behavior of children with autism, while effectively improving their language skills, social skills, and play skills [6]. Therefore, instructional interventions to address common attention deficits in children with autism can be beneficial to the development of common attention, as well as improving other related skills [7, 8].

The contributions of this article are as follows.

We explored whether the combined orientation model of DTT and PRT can improve the joint attention ability of children with autism. Using the cross-behavior multiexploratory design in the single-subject research method, two preschool children with autism were selected as subjects, and the independent variable was shared attention teaching.

Based on the behavioral performance of the constituent elements of common attention, this research provides operational definitions for each subgoal of common attention, enriching the empirical research on common attention of children with autism and provides the methods and suggestions of common attention intervention research for autistic children.

The intervention model of this study is taken from the joint attention intervention plan. The researcher and the children conduct one-to-one joint attention training in a training room, and the time is about 5–8 minutes. Adopt DTT teaching principles and train joint attention by systematically prompting the level.

## 2. Related Work

The developmental response orientation is a consistent and natural way of developing joint attention, which helps to develop joint attention, following the child's attention; play and interest help to promote eye contact; responding to the child's associative communication behavior in a timely manner promotes the frequency and efficacy of mutual communication, and using multiple cues allows the child to pay more attention to adult attentional cues. Reference [9] collated current JA intervention programmes and concluded that the orientation of the programme can be divided between naturalistic teaching and single-attempt training, where the naturalistic teaching orientation is similar to natural parent-child interaction, and the single-attempt training orientation requires the child to respond correctly to stimuli provided by the adult and to practice the target behavior extensively [10]. Research collating interventions related to joint attention can be divided into four orientations: the single-attempt training orientation, the developmental-responsiveness orientation, the communication-support orientation, and the combined approach (combined approach). Reference [11] provided children with cues so that they can perform the target behavior, as well as repetitive exercises, in a process that is primarily adult-led instruction. The results of the study showed an increase in the frequency of all postural and oral responses but were not consistent with the aim of shared attention and could not be analogous to natural contexts [12]. Using applied behavioral analysis, teaching was divided into components including, first, table training time using DTT, second, floor time, using something the child is interested in and following the child's lead, and, third, random teaching of target behaviors. Reference [13] suggested a three-point teaching approach where the instructor uses imitation of the child's behavior without using prompts to engage the child, the instructor moves their face and objects of interest to the child to get the child's attention, the intervention focuses on social awareness, and the sequence of development is eye contact, noticing an adult partner, taking turns, engaging behavior, spontaneous requests, and nonverbal shared attention.

Using a developmental orientation, [14] used eye contact and active display with young children as teaching goals. After the intervention, children showed a significant improvement in the target behavior, but spontaneous joint attention was poorer in terms of effectiveness and authorisation. Reference [15] divided the instructional content into a 5-stage intervention process and taught imitative behavior to young children with autism. The SCERTS model developed by [16] refers to seven intervention principles, including an emphasis on the functional use of language and communication in all natural contexts; consideration of the child's emotional regulation and its impact on communication, social interaction, and learning; and the integration of behavioral problems into social communication training programmes and the analysis of behavioral functioning and positive behavioral treatment. Reference [17] combined DTT orientation and PRT teaching interventions to improve joint attention in children with autism and found that both children showed progress in joint attention after the intervention; [18] mainly referred to an intervention programme that divided the training process into tabletop and floor time, with the therapist and parents as the intervenor, and analysed behavioral records from the intervention process; [19] conducted a joint attention intervention with a child with autism. A joint attention intervention with an integrated table and floor time resulted in an increase in both target behavioral skills for this child. Reference [20] used psychoanalytic linguistics, behavior management techniques, and a social-pragmatic orientation to guide parents in teaching their young children with ASD at home (mean age: 21.4 months), with the goal of increasing the routine of joint activities and directly teaching joint attention. Reference [21] combined a core response training with a communicative-supportive orientation and DTT training with a single-attempt orientation. Following behavioral routines, cues that teach children a response-attention orientation are also known as response-based joint attention training.

## 3. Knowledge Background

Joint attention is one of the earliest social behaviors in children and is a foundation for the development of language and interpersonal interactions. Deficits in joint attention are one of the core deficits of children with autism, and improving joint attention in children with autism can help improve the development of nonverbal and verbal expression, social initiative, and emotional control in children with autism. This study proposes implementing an intervention for children with autism in a natural developmental setting as a way to improve joint attention in children with autism. The effectiveness of the teaching methods and interventions used in this study can effectively promote the application of information technology for joint attention interventions, and the methods used in the study are convenient and effective, with strong practical operational implications [22].

### 3.1. DTT

Discrete Trial Teaching is an approach of teaching that uses applied behavioral analysis as a core principle [23]. Each instruction has a clear beginning and ends. After becoming familiar with each small part of the technique, further stimuli are presented. The teacher makes demands on the student to obtain a response, needs to guide the student to produce the appropriate behavior, and gives immediate and timely positive feedback when the correct response is required.

### 3.2. PRT

Discrete Trial Teaching proposes critical response training based on the characteristics associated with learning in children with autism, which is taught through a “stimulus-response-consequence” approach, supported by positive behavior and emphasising unstructured situations. This approach uses “stimulus-response-consequence” teaching, supported by positive behaviors and emphasising unstructured situations to help children learn core skills [24]. Core areas for change through PRT interventions are as follows: increasing self-initiated motivation, teaching children how to respond to learning and social interaction opportunities in natural contexts, reducing the need for constant supervision by intervention strategy providers, and reducing the need to remove children from natural contexts.

### 3.3. Shared Attention

Joint attention (JA) is the basis of cognition and emotion and is a preverbal communication skill [25]. Discrete Trial Teaching suggests that normal children have nonverbal social interactions between themselves and others almost from birth and that, in early communication, young children communicate with partners through joint attention, sharing things of common interest with them. In early communication, children communicate with their partners through joint attention, sharing things of common interest with them, which is a form of joint attention that involves the child, others, and objects.

To sum up, joint attention means the three following things: (1) Focus of attention: joint attention is a three-person relationship that requires two subjects which connect with each other through some externally visible behavior; that is, two subjects have a common focus of attention on events (including people, things, and objects) at the same time. (2) Triggering subject: the different triggering subjects can be divided into responding joint attention and behavioral manifestations, which can include eye contact, close (distant) instruction following, and active display. (3) Purpose: the purpose of joint attention is to share socially rather than to satisfy individual needs.

## 4. Strategies for Joint Attention Intervention for Children with Autism

In reference to national and international research, these three main strategies for communist interventions were found. Common attention intervention strategies are divided into Natural Environment Teaching, Play Oriented Teaching Intervention, and SCERTS Model Intervention models. The following are descriptions of each model.

### 4.1. Teaching Interventions in the Natural Environment

Discrete Trial Teaching proposes the milieu teaching approach. Discrete Trial Teaching states that children's initiative in the presence of something interesting, something they enjoy, or an activity, increases and they become actively involved. Thus they actively participate in it. The four strategies of demonstration, prompting-demonstration, time delay, and random teaching are briefly described in Tables 1 and 2.

The table shows that teaching interventions in the natural environment emphasise functional developmental learning in the natural environment, the importance of spontaneous learning and authorisation, and the use of demonstration, prompting-demonstration, time delay, and random teaching strategies in the process of teaching interventions in the natural environment.

### 4.2. Play and Culture Intervention (PCI)

A broad intervention strategy is designed using a playful approach, based on developmental theory and supported by behaviorist, cognitive, and social constructivist theories. The aim is to promote social competence and communication in a natural environment for children with autism. Continuing with the previous play-based educational design, Play and Culture Intervention (PCI) is a Taiwanese intervention model for children with autism [26]. The connotations of Play and Culture Intervention are, firstly, to improve the autistic children's skills in learning culture on their own, secondly, to build a platform for children's learning abilities through social interaction and play and knowledge of daily life, thirdly, to allow children to learn the essence of local civilization, and, fourthly, to build a platform for mutual support so that children can learn cultural knowledge.

Play and Culture Intervention model therefore places particular emphasis on interventions in everyday life, for example, food, clothing, housing, transport, and play. However, in everyday life, children with autism have various learning difficulties due to nourishing characteristics such as inability to concentrate, lack of intrinsic motivation, discomfort with sensory regulation, and other personal reasons, as well as objective reasons such as the environment they are in being too noisy and the short duration of the intervention, so it is necessary to intervene in cultural knowledge through play.

The combination of Play and Culture Intervention, based on the child's own culture, following the child's interests, and using the routines of the natural environment as a choice of environment and context for interventions, can be very helpful in the development of spontaneous learning skills or in the development of categorization.

### 4.3. Intervention Model

The intervention model in this study was taken from the common attention intervention programme, the combined orientation mentioned earlier, where the first half of the intervention was taught by DTT and the second half by PRT.

One-to-one joint attention training was conducted by the researcher and the child in an individual training room for approximately 5–8 minutes. The principles of DTT were used to train joint attention through systematic cueing levels.

PRT teaching continues the DTT teaching training of joint attention, emphasising the enhancement of joint attention states. The process places emphasis on positive affective communication, following the child's lead, waiting for the child to initiate play, not forcing to necessarily start to play or participate in activities, and providing encouragement when the child is having difficulties or needs help. The study on training shared attention behavior in young children with autism mentioned that all situations during floor time were manipulated and set up with the intention of promoting socialization and communication in young children.  Table 3 shows interactive strategies for teaching PRT.

## 5. Shared Attention Teaching Effectiveness

### 5.1. Effectiveness of Subject A's Teaching

This subsection focuses on the graphs of the effects of teaching the three target behaviors of subject A and the results of the visual analysis between the stages, as illustrated below for the immediate and sustained effects of teaching the three joint attentional behaviors of eye alternation, following instructions, and active display.

As can be seen in Figure 1, during the baseline period, subject A performed poorly on all three skills of the target behavior. With the joint attention intervention, subject A's scores on the three target skills were significantly higher than those in the baseline period, indicating that the joint attention intervention had an immediate effect on subject A. During the maintenance period, subject A's scores for eye contact and following instructions also remained above 80, indicating a maintenance effect on the learning of eye contact and following instructions.

The study used percentage graphs to visualise the results of the data. As can be seen from the graph, the subjects' eye alternating behavior increased during the intervention period relative to the baseline period. The frequency of their eye alternating behavior was also higher and increasing in the maintenance period compared to the baseline period. Therefore, it can be tentatively determined that joint attention instruction was effective in intervening in subject A's eye alternating behavior and that it was somewhat effective in maintaining it.

As can be seen from Figure 2 and Table 4, during the four observations in the baseline period, the percentage of correct performance of the “eye alternation” target behavior by subject A was 0, showing a stable state, indicating that subject A had not mastered the target behavior prior to entering the intervention period. During the six observations recorded during the intervention period, the percentage of subjects' eye turnover target skills ranged from 50% to 80% during this period, with the mean percentage of the period increasing from 0% to 73.33%, showing an upward trend and a stable level during the latter part of the intervention period. The change in level was +30%, with a positive trend, indicating that the intervention was more effective during the intervention period, with subject A showing teaching effectiveness at the first postintervention rating, with the percentage achievement of the eye alternation increasing to 50% and reaching a stable 80% at the third to sixth rating. During the maintenance period, 11 sessions were recorded, with a tendency towards stability of 50%, which is variable, a level range of 80%–90%, and a level change of 0%, which is a stable level of 83.3%. This indicates that DTT combined with PRT had a significant effect on the autistic child's joint attention target behavior [27].

Table 5 shows that the learning behavior of subject A's eye alternation, between the two phases from the baseline period to the intervention period, the trend path from level to rise, is in a positive effect change, with an interlevel change of 50%–0%, and the overlap between the baseline and intervention periods is 0%. The trend path and increase in level from the baseline and instructional periods show that subject A's eye alternation behavior improves significantly after the instructional intervention. The dry expectation is followed by the maintenance period. In this stage, the change between trend effect levels is 10%, and the overlap between dry expectation and maintenance period is 9%.

In summary, it can be s7een that joint attention teaching has a significant and consistent effect on eye alternation in cases of joint attention.

As can be seen from Figure 3 and Table 6, the mean percentage of correct performance of the target behavior in the baseline period was 5%, indicating that subject A had not mastered the target behavior before entering the intervention period. Over the 5 observations recorded during the intervention period, the percentage change in the range of subject A's indicator following target level during this period ranged from 60% to 90%, with the mean percentage change during the period increasing from 5% to 82%, showing an upward trend and a stable level during the latter part of the intervention period. The change in level was +40%, with a positive trend, indicating that the intervention was more effective during the intervention period, with subject A showing instructional effectiveness at the first postintervention rating, with the percentage of instructional following achieved increasing to 50% and reaching a stable effect of 90% at the third to fifth rating. During the maintenance period, there were 10 recordings, with a tendency towards stability of 80%, a range of 90%–90% and 0% change in level, and a level of stability of 80%. This indicates that DTT combined with PRT had a significant effect on the autistic child's joint attention target behavior.

As seen in Figure 4, the mean percentage of subjects who correctly performed the “active display” target behavior during the four observations in the baseline period was 0%, showing a stable state, indicating that subject A had not mastered the target behavior before entering the intervention period. Over the 6 observations recorded during the intervention period, the percentage change in the range of subject A's active display of the target behavior during this period was 40%–60%, with the mean percentage change during the period increasing from 0% to 51.7%, showing an upward trend and a stable level during the latter part of the intervention period. The change in level was +20%, with a positive trend, indicating that the intervention was more effective during the intervention period, with subject A showing teaching effectiveness at the first postintervention rating, with an increase in the percentage of active displays achieved to 50% and a positive and stable effect from the second rating to the sixth rating. In summary, subject A's following instructions was achieved at a higher rate during the intervention period than during the baseline period, and the percentages remained stable and high during the maintenance period, suggesting that DTT combined with PRT had a significant effect on this child's joint attention target behavior.

### 5.2. Effectiveness of Subject B's Teaching

This subsection focuses on the graphs of the effects of teaching the three target behaviors and the results of the interstage visual analysis for subject B. The following is a description of the immediate and sustained effects of teaching the three coattentive behaviors of eye alternation, following instructions, and active display for subject B.

As can be seen in Figure 5, subject B performed poorly on the three target skills of eye alternation, following directions, and active display during the baseline period. All three target skills were underperformed by subject B during the baseline period. Subject A's score on the three target skills was significantly higher than that at baseline. This indicates that the joint attention intervention had an immediate effect on subject B. During the maintenance period, subject B scored significantly higher on the three target skills than at baseline, indicating that the joint attention intervention had an immediate effect on subject B. In the maintenance period, subject B also maintained scores above 80 in eye alternation and following instructions, indicating a maintenance effect on the learning of the two target skills of eye alternation and following instructions.

A line graph was used to visualise the results of the data. The graph shows that subject B showed an increase in eye alternating behavior in the intervention period compared to the baseline period. During the maintenance period, the frequency of eye alternating behavior was also higher than that during the baseline period and was increasing. Therefore, it can be tentatively determined that joint attention instruction was effective in intervening in subject B's eye alternating behavior and that it was somewhat effective in maintaining it.

As seen in Figure 6, the mean percentage of correct performance of the “eye alternation” target behavior for subject B was 0% for the four observations recorded during the baseline period, showing a steady state, indicating that subject B had not mastered the target behavior before entering the intervention period. Over the 6 observations recorded during the intervention period, the percentage change in the range of the subject's active display of the target skill during this period was 20%–80%, with the mean percentage change during the period increasing from 0% to 66.7%, showing an upward trend and a stable level during the latter part of the intervention period. The change in level was +60%, with a positive trend, indicating that the intervention was more effective during the intervention period, with subject B showing teaching effectiveness at the first postintervention evaluation, with the percentage of achievement increasing to 50% for the eye alternation and reaching a stable effect of 80% from the third to the sixth evaluation.

As seen in Figure 7, the mean percentage of correct performance of the “follow the instructions” target behavior for subject B was 0% for the four observations recorded during the baseline period, showing a stable state, indicating that subject B had not mastered the target behavior before entering the intervention period. During the six observations recorded during the intervention period, the percentage change in the range of the subject's following the instructions target skill level during this period was 60–80%, with the mean percentage change during the period increasing from 0% to 73.3%, showing an upward trend and a stable level during the latter part of the intervention period. The change in level was +20%, with a positive trend, indicating that the intervention was more effective during the intervention period, with subject B showing instructional effectiveness at the first postintervention assessment, with an increase in the percentage achievement of the following instructions to 60%. During the maintenance period, there were 6 recordings with a range of 70%–90%, a 10% change in level, an 80% trend towards stability, and a 100% level of stability. In summary, the percentage of target behaviors achieved during the intervention period was significantly higher than that during the baseline period, and the percentage of instructions followed during the maintenance period was also higher than that during the baseline period, suggesting that DTT combined with PRT had a significant effect on the child's joint attention target behaviors and that the maintenance period maintained the same level of behavioral achievement as the intervention period.

As can be seen in Figure 8, the mean percentage of the target behaviors that were correctly performed by subject B during the four observations in the baseline period was 0%, showing a steady state, indicating that subject B had not mastered the target behaviors before entering the intervention period. Over the 6 observations recorded during the intervention period, the percentage change in the range of the subject's active display of the target behavior during this period was 40%–60%, with the mean percentage change during the period increasing from 0% to 55%, showing an upward trend and a stable level during the latter part of the intervention period. The change in level was +20%, with a positive trend, indicating that the intervention was more effective during the intervention period, with subject B showing teaching effectiveness at the first postintervention assessment, with an increase in the percentage of active demonstration achieved to 50%. During the maintenance period, there were 6 recordings with a range of 70%–90% and a 20% change in level during the period, with a tendency towards stability and a level of stability of 80%. In summary, the percentage of target behaviors achieved during the intervention period was significantly higher than that in the baseline period and the percentage of active displays achieved during the maintenance period was also higher than that in the baseline period, indicating that DTT combined with PRT had a significant effect on the child's joint attention target behaviors and that the maintenance period maintained the level of behavior achieved during the intervention period.

## 6. Conclusions

The aim of this study was to investigate whether the use of a combined orientation model of DTT and PRT could improve joint attention skills in children with autism. The study used a cross-behavioral multitest design in a single-subject research method, with two preschool children with autism as subjects, with the independent variable being joint attention instruction and the dependent variable being the three joint attention skills. DTT combined with PRT instruction improved joint attention in children with autism. After the instructional intervention, children with autism showed a significant increase in correct “eye alternation,” “following directions,” and “active display” behaviors.

## Figures and Tables

**Figure 1:** Plot of percentage achievement of the three target behaviors for subject A.

**Figure 2:** Percentage of subject A's eye alternations achieved.

**Figure 3:** Percentage of subject A's eye alternations achieved.

**Figure 4:** Plot of the percentage of active displays achieved by subject A.

**Figure 5:** Plot of percentage achievement of the three target behaviors for subject B.

**Figure 6:** Percentage of subject B's eye alternations achieved.

**Figure 7:** Graph of percentage of following instructions achieved.

**Figure 8:** Proactive display reach percentage graph.

**Table 1:** Description of the content of the four strategies of demonstration, prompting-demonstration, time delay, and random teaching.

Strategy	Content
Demonstration	In the teaching process, it is child-centered and combined with the environment. In the teaching process, there are specific teaching aids, teaching postures, and teaching contents for children to imitate or follow and repeat.
Tips-demonstration	In the process of teaching, the teacher asks the children to wait systematically or delay for a short time before giving assistance, so as to encourage children to actively interact.
Time delay	In the process of teaching, the teacher asks the children to wait systematically or delay for a short time before giving assistance, so as to encourage children to actively interact.
Random teaching	The purpose is to trigger more complex language types and higher language skills for specific subjects, so as to improve the ability of conversation and prolong the time to talk about the subject.

**Table 2:** DTT teaching system prompt level table.

Children's behavior	Prompt level used	Example
Early learning No target behavior at all	6: combining language and whole body tips	The child took away the toys on the table. The teacher held the child's toy hand up to his eyes and said, “show it to me.”

Slightly partial target behavior	5: combining language and some body tips	The child picked up the toy and stretched it in the direction of the teacher but did not raise it. The teacher gently pushed the child's hand to remind him to raise it to his eyes and said, “show it to me.”

In the middle of learning, the strength of using some body tips becomes smaller. Children seem to understand that the teacher requires them to perform a certain action first after they get the toy	4: language prompt accompanying demonstration	When the teacher touches the child's elbow, he can lift it up to his eyes. The teacher also lifts the toy up to the child's eyes and says, “you see, I have this (toy).”
	3: special language tips	When the teacher touches the child's elbow, he can lift it up to his eyes. When the child picks it up and extends it to the teacher, he says to the child, “show it to me.”

At the later stage of learning, children can stably show target behavior under the hint of level 3	2: general language tips	When the children got the toys on the table, the teacher said, “what did you get?”

Children can stably show target behavior under the hint of level 2	1: unguided physical space tips	When the child gets the toy on the table, the teacher puts his face forward to remind the child to raise it for others to see.

**Table 3:** PRT teaching and learning interaction strategies.

Interactive strategy	Explain
*Basic interaction strategy*	
Follow the lead of children	Understand children's hobbies, observe, and wait
Say what the child is doing	Short and clear instructions. Put the ball in
Repeat what the child said	Repeat the words or pronunciation

*Environmental regulation strategy*	
Sit close to the child and make eye contact	Accompany them
Adjust the environment to make it suitable for children's games	For example, put their favorite things in an easy to take place
Help but not help	For example, if the bag cannot be torn open, you can help him tear a small opening and let him finish the rest by himself

*Interactive response strategy*	
Expand what children say	For example, when children say “horse,” it can be extended to “horse is eating grass”
Correct feedback	Encourage and enhance children's behavior towards children, and stop children's destructive or dangerous behavior
Fun of manufacturing activities	Add sound effects to the activity or do not respond as expected

**Table 4:** Summary table of statistical analysis within the eye alternation phase.

Stage	Baseline period	Intervention period	Holding phase
Stage length	4	6	11
Trend stability	Stable 100%	Unstable 50%	Stable 100%
Leveling range	0	50%–80%	80%–90%
Horizontal stability	Stable 100%	Stable 100%	Stable 100%
Level change	0	83.3%	10%

**Table 5:** Summary table of statistical analysis between phases of eye alternation.

Phase comparison	Intervention period/baseline period	Maintenance period/intervention period
Trend effect	Forward	Forward
Trend stability	Stable to unstable	Unstable to stable
Variation between levels	50%–0%	90%–80%
Average level change	73.3%	15.97%
Overlap percentage	0	9%

**Table 6:** Summary table of statistical analysis within the indicative following phase.

Stage	Baseline period	Intervention period	Holding phase
Stage length	4	5	10
Trend stability	Unstable 50%	Stable 80%	Stable 100%
Leveling range	0%–20%	60%–90%	90%
Horizontal stability	Unstable 75%	Stable 80%	Stable 100%
Level change	20%	30%	30%

## Data Availability

Analytical permission was not obtained from the data provider because of trade confidentiality.
